This article has been retracted.

# An evaluation of the potential consequences of drilling titanium and tantalum implants during surgery - a pilot study

**DOI:** 10.1186/s12891-017-1784-x

**Published:** 2017-11-03

**Authors:** Paweł Skowronek, Paweł Olszewski, Wojciech Święszkowski, Marcin Sibiński, Marek Synder, Michał Polguj

**Affiliations:** 1 Clinic of Orthopedic and Traumatology, Regional Hospital and Kochanowski Medical University, Kielce, Poland; 2 Faculty of Materials Science and Engineering, Warsaw University of Technology, Warsaw, Poland; 3 Clinic of Orthopedics and Pediatric Orthopedics, Medical University of Lodz, Lodz, Poland; 4 Department of Angiology, Medical University of Łódź, ul. Narutowicza 60, 90-136 Łódź, Poland

**Keywords:** Hip arthroplasty, Knee arthroplasty, Augments, Revision, Loosening, Drilling

## Abstract

**Background:**

The aim of the study was to evaluate the potential consequences of drilling titanium alloy (Ti) and tantalum (Ta) implants.

**Methods:**

During an in vitro study, four holes were made in each of two spatially porous trabecular implants: one Ta and the other Ti alloy (Ti-6Al-7Nb). The weight and the volume of particles produced during the drilling were then measured using a Radwag XA 110/2X (USA) laboratory balance.

**Results:**

The loss of mass of the Ti and Ta implants was respectively 1.26 g and 2.48 g, and the volume of free particles was respectively 280 mm^3^ and 149 mm^3^. The particles were recovered after each stage. Despite the use of 5 μm filters, around 0.6% of the total implant mass from both implants was not recovered after drilling (roughly 2% of the mass of the particles created).

**Conclusion:**

It is technically difficult to make holes in Ti and Ta implants using standard surgical tools, and the process creates a significant amount of metal particles which cannot be removed, despite intensive flushing. This may have a potentially adverse influence on the survival of the implant and result in negative systemic consequences.

## Background

The reconstruction of joints with revision augments is gaining popularity as a method of enabling the replacement of bone tissue through the metal elements, thus allowing osteointegration of the bone tissue with the implant. Currently, orthopaedic surgery employs implants which use various methods of maintaining a porous outer structure; the most common being hydroxyapatite coatings and trabecular metal implants, which have a spatially porous architecture that allows bone tissue to heal within the implant. The most commonly used implants are made from such materials as tantalum or titanium and its alloys [1–9].

At the macroscopic level, various kinds of spatial elements can be used to permit the partial alignment of bone defects. Such elements can be combined with each other and with bone tissue. Most have already been provided with holes for titanium screws to allow primary stabilization. These elements are usually connected to each other using polymethyl methacrylate (PMMA), a bone cement, or they can be joined mechanically using screws [2, 3, 10]. This porous tantalum biomaterial has shown to have very good characteristics for bone ingrowth [10, 11]. Unfortunately, the creation of standardized holes does not always offer full potential stability for the implant in bone tissue; this requires the creation of additional holes in the implant or risks damage to the metal structure of the implant while testing the mechanical stability of two or more metal elements. During procedures performed in our own surgical practice, difficulties have often been encountered in creating stable external augments with standard holes, even with good pre-operative planning. Hence, the question arises whether drilling porous titanium or tantalum augments is safe for the patient and may potentially compromise implant stability.

During the mechanical production of the implant, many small metal particles are created; these may have a significant impact on the survival rate of the implant and its secondary stabilization, hasten its wearing and may loosen the node elements of the tribological endoprosthesis. The release of macroscopic and microscopic particles can also ultimately lead to osteolysis and metalosis of the tissues. In vitro studies have also reported necrotic effects to be associated with the fibroblast [12, 13].

The aim of the study was to evaluate the potential consequences of drilling titanium alloy (Ti) and tantalum (Ta) implants. No similar studies were identified by a review of extant literature.

## Methods

This in vitro study used two trabecular implants made from spatially porous materials, one from tantalum, and the second from titanium alloy (Ti-6Al-7Nb) (Zimmer, USA). The tantalum implant has a consistent 3D tantalum structure similar to cancellous bone and up to 80% porosity. Its average pore size is of 440 μm, has low modus of elasticity and a 0.98 coefficient of friction for net shape parts. The titanium implant also has a 3D structure. Its porosity is 67% and strength (extendibility) < 40 MPa [14]. The standard orthopaedic titanium and tantalum samples had a height of 10 mm. In each material sample, four holes were made to the full depth of the twist drill with a diameter of 4.5 mm. (BBrown Aesculap, Germany Tuttlingen). This drill diameter is one of the standard drill diameters used in orthopaedic surgical procedures of the knee.

Before the holes were made, the volume of the individual implants was measured as well as their mass. Initial attempts were made using a standard drill used for bone tissue. A drill press was used to make the holes. Unfortunately, after a 10 min drilling period, with the hole being cooled with 0.9% NaCl aqueous solution, only holes of 2 mm depth were obtained in each implant material, without the possibility of drilling all the way through. Using this technique, more than 200 ml of fluid with metal elements was obtained, which under in vivo conditions, may remain in the bone tissue and surrounding soft tissues.

After changing drill bits for one with a sharp cobalt carbide bit, it was possible to make through-holes in the samples of both implant materials. The use of a bit tipped with carbide cobalt shortened the time to drill each hole to approximately 25 s, and this time was similar for both materials.

Next, the volume and weight of the particles created in the drilling process were measured. During the drilling operation, saline was used to cool the drill bit. After all the holes were created, all material derived from the drilling process was collected. Then, any additional material remaining within the 3D structure of the Ti alloy and Ta implants was collected by further washing with distilled water using an ultrasonic bath. The volume and weight of the individual sizes of the metal particles were obtained by filtration, by running both the saline and distilled water through filter papers with reducing pore sizes. All samples were weighed using Radwag XA 110/2X (USA) laboratory scales with an accuracy of 0.01 mg. The volume of the obtained “fines” was measured by titration using a 10 mm^3^ measurement system.

The study had been approved by the Bioethical Committee of the Medical University of Łódź, Poland and followed the rules of the Declaration of Helsinki.

## Results

The loss of mass of the implants was measured, as was the volume and size of the particles obtained while drilling the through-holes. The loss of mass of the titanium implant (1.26 g) was approximately half that of tantalum (2.48 g) (Fig. 1). However, the volume of free particles created by the drilling of the titanium implant (280 mm3) was nearly twice that of the tantalum implant (149 mm3) (Fig. 2).

**Fig. 1:** Weight loss of implants: Titanium (Ti) and Tantalium (Ta)

**Fig. 2:** The volume of the recovered tantalum and titanium particles from drilling the titanium (Ti), and tantalum (Ta) implants

The first evaluation of the proportion of free particles was obtained from the NaCl solution used as a cooling fluid during drilling; both macroscopic and microscopic particles were present in the fluid. In this transfer stage, an ultrasonic system was used with a filter diameter of 200 μm. In total, 67.83% (titanium alloy) and 68.43% (tantalum) of all particles produced as a result of drilling were obtained from the fluid.

The second wash in distilled water using an ultrasonic bath recovered an additional 29.20% of the entire volume of implant particles for titanium alloy and 13.91% for tantalum. In this stage, the filter diameter was 50 μm. Finally, after the implant was cooled, the smallest filter with the diameter of 5 μm was used. An additional 0.4% of total particle volume was obtained from the titanium alloy and 9.32% from the filtrate after rinsing the implant, and 0.56% of the volume of particles of titanium alloy and 6.37% loss in volume of implants for tantalum material particles (Fig. 3). About 0.6% of the entire weight of the implants before drilling (about 2% by weight of the particles created by drilling) was not recovered after drilling, despite the use of 5 μm filters.

**Fig. 3:** The percentages of recovered titanium (Ty), and tantalum (Ta) after drilling implants and the use of measurements for the different stages of the recovery of the particles with saline (NaCl) and distilled water (DW)

## Discussion

Highly porous tantalum designs are known to have good mechanical properties and have been shown to exhibit superior stability to traditional cementless acetabular implants [2]. The greater potential for bone and fibrous ingrowth demonstrated by tantalum may be related to its porosity, which is approximately two to three times greater than that of cobalt, chromium or titanium mesh [10, 11]. Those implants have several additional advantages: the modulus of elasticity of porous tantalum is similar to that of subchondral bone, allowing greater physiological transfer of load to the host bone; in addition, they are stronger than structural allografts, and have a higher coefficient of friction than traditional cementless designs, resulting in better stability [1–3]. These properties allow these implants to be used in modern orthopaedics in difficult primary and revision hip and knee arthroplasties, foot and ankle surgery or dental implants [4–8]. Trabecular metal implants have also been awarded higher scores in selected arthroplasties than conventional components [9].

The aim of the present study was to identify the potential consequences of drilling holes in Ti alloy and Ta implants. In addition to the difficulties associated with creating holes in the tested implant materials, there is a high risk of leaving particles of implant material in the living tissue. Despite intensive washing under laboratory conditions, it was not possible to remove all the free particles created while drilling the material and avoid damage to the implant. The effectiveness of the removal of metal particles would arguably be much less when performed in the operating room, resulting in even more particles remaining in the tissues of the patient. Twice the volume of particles were left by the titanium alloy implant than the tantalum implant. Also, a greater amount of the smallest particles were left behind when tantalum was used, with an associated greater risk of them entering the blood vessels.

Hence, intraoperative interference with the structure of both tantalum and titanium implants may be detrimental to the patient [12, 13, 15]. It can also shorten the biofunctionality of the prosthesis and lead to systemic effects. Leaving particles of titanium alloy or tantalum behind after drilling can increase the risk of faster wear of the surface polymer or ceramic inserts and the tribological head node of the prosthesis, and can increase the risk of bone disease, especially around the cup, consequently shortening the functional lifetime of the prosthesis [15]. Furthermore, small particles of metal particles including Ti and Ta particles has been shown to cause fibroblast necrosis in in vitro studies [12, 13]. Mostardi et al. found cell death to occur equally for both metals, and that its degree was related to the size and concentration of the particles produced rather than the type of metal tested [13]. Small metal particles can pass through the cell plasma membrane and enter the blood stream mainly by diffusion or endocytosis [16]. Diffusion can occur directly or through membrane channels, and conveys metal nanoparticles measuring 200 nm or smaller, with a preference for those of 50 nm [16, 17]. Larger fragments are taken up by phagocytic processes of specialized cells such as macrophages [18].

An additional problem may be associated with the increase in biotoxicity associated with released particles of niobium, vanadium and aluminum present in the titanium alloy implants. It seems that despite leaving behind a greater mass of metal shavings in the patient, the Ta implants may in fact be less harmful, insofar that they do not subject the patent to any elevated risk of biotoxicity, type I or IV allergy or risk of accumulating rare metals in the CNS [19, 20]. In the case of the titanium implants, twice the number of metal ions remained, particularly vanadium and niobium, which results in a greater risk of negative biological impact. Despite intensive rinsing it was not possible to fully remove the remaining metal particles created while drilling the holes. In the case of tantalum, a greater number of smaller particles were left in the operating field, with a greater risk of absorption into the blood. Regarding the use of tantalum without the use of niobium or aluminum, the toxicity of the remaining tantalum ions should be less than with Ti-Al-Ni or Ti-Al-V alloys [19–21]. Therefore we predict that interoperative drilling in the implant of the structure, particularly those constructed from of alloys of different metals, may have detrimental effects for the patient: it can result in increased chance of nephrotoxicity, ion accumulation in the central nervous system and the possibility of allergy. This mainly applies to alloys with vanadium and niobium [19–21].

In our opinion, it is not recommended that additional holes be created in Ta and Ta augments in everyday surgical practise. It is impossible to remove drilling products by passive and pressure washing in a laboratory setting, and in the operating area it would be not possible even with the use of lavage systems. In addition, it is impossible to drill holes in the implants with standard bone drills, and carbide drill bits that could be used for medical purposes are rarely available in operative surgery: no suitable supplier could be found in our country.

As similar articles could not be found in the literature, it is difficult to compare the results of our study with others. This is intended as a pilot study which will be continued in the future to gain results that will be suitable for statistical analysis.

## Conclusions

The creation of openings in Ti alloy and Ta implants is a technically difficult operation when performed using standard surgical tools, and results in the creation of a significant amount of metal particles, which cannot be removed, despite intensive flushing. This may have a potential adverse influence on the survival of the endoprosthesis and have negative systemic consequences.

## Abbreviations

PMMA: Polymethyl methacrylate
Ta: Tantalum implant
Ti: Titanium implant
